# The Effects of Transcutaneous Acupoint Electrical Stimulation on Cancer-related Fatigue and Negative Emotions in Cancer Patients: A Systematic Review and Meta-Analysis of Randomized Controlled Trials

**DOI:** 10.1155/2022/1225253

**Published:** 2022-07-31

**Authors:** Yubo He, Minchi Yuan, Chun He, Danwei Zhu, Feida Wang

**Affiliations:** ^1^Department of Rehabilitation Medicine, The First People's Hospital of Jiashan/Jiashan Branch of the Second Affiliated Hospital of Zhejiang University School of Medicine, Jiaxing, China; ^2^Department of Oncology, The First People's Hospital of Jiashan/Jiashan Branch of the Second Affiliated Hospital of Zhejiang University School of Medicine, Jiaxing, China; ^3^Department of General Medicine, The First People's Hospital of Jiashan/Jiashan Branch of the Second Affiliated Hospital of Zhejiang University School of Medicine, Jiaxing, China; ^4^Department of Traditional Chinese Medicine, Tongde Hospital of Zhejiang Province, Hangzhou, China

## Abstract

Transcutaneous electrical acupoint stimulation (TEAS) is a noninvasive and therapeutic technique that stimulated the acupoint by delivering electricity. Whether TEAS could relieve cancer-related fatigue (CRF), anxiety, and depression and improve the quality of life in cancer patients remains controversial. Thus, we conducted a thorough literature search of electronic Chinese and English databases for randomized controlled trials (RCTs) reporting the effect of CRF, anxiety, depression, and quality of life in cancer patients from inception to July 1^st^, 2021. The Cochrane Collaboration Risk of Bias criteria were used to assess the risk of bias for each included RCT. Continuous variables were analyzed using standardized mean difference (SMD) and 95% confidence interval (CI). A fixed-effects model was used for the meta-analysis of all outcomes. A total of nine RCTs with 924 cancer patients were included in this analysis, including 460 patients in the interventional group and 464 patients in the control group. We found that TEAS could significantly reduce CRF, depression, and anxiety (SWD = −0.83, 95% CI: −0.99 to −0.66, *P* < 0.05) and improve the quality of life (SWD = −1.37, 95% CI: −2.34 to −0.40, *P* < 0.05). The funnel plot analysis revealed no significant publication bias. We conclude that TEAS is beneficial for reducing CRF, depression, and anxiety and improving the quality of life of cancer patients, but additional high-quality evidence in the future is entailed to support this.

## 1. Introduction

Tumor cells can be eliminated through a variety of methods, including surgery, chemotherapy, radiotherapy, molecular targeted therapy, and immunotherapy [1]. However, most of these treatments are associated with significant side effects. For instance, 30–60% of cancer patients undergoing treatment reportedly develop severe cancer-related fatigue (CRF), which can lead to treatment interruption because of poor results from reduced physical function and reduced motor capacity [1]. Fatigue usually decreases within a year after treatment completion, but CRF is expected to last for months or even years in a small subset of patients after successful treatment [2]. In addition, cancer patients may develop serious negative emotions such as depression and anxiety, which further adversely affect the overall quality of life.

Transcutaneous electrical acupoint stimulation (TEAS) is a noninvasive therapeutic approach based on percutaneous electrical nerve stimulation [3]. TEAS uses a combination of electrodes with traditional Chinese acupuncture to stimulate specific acupoints of the body without needles, relieving symptoms and facilitating recovery [3]. Currently, the clinical application of TEAS in cancer patients and those with negative emotions remains controversial. Hou et al. [3] reported that the Revised Piper Fatigue Scale (RPFS) scores of the interventional group decreased significantly compared with the control group after 28 days of TEAS treatment for lung cancer, indicating that TEAS may help reduce the CRF in lung cancer patients. However, there was no statistical difference in the RPFS scores between the interventional and control groups in terms of the effect of TEAS on CRF in breast cancer patients [4]. The therapeutic effects of TEAS on CRF, negative emotions, and quality of life of cancer patients remain largely unknown. Therefore, our review aims to systemically analyze and study on the effect of TEAS in cancer patients and to quantify the effects of TEAS.

## 2. Methods

### 2.1. Search Strategy

Investigators searched for eligible literature from the following electronic databases: PubMed, Web of Science, Embase, Cochrane Library, China National Knowledge Infrastructure (CNKI), Chinese Biomedical Literature Database (CBM), Wanfang Database, and Chinese Science and Technology Journal Database (VIP). For example, we searched PubMed using combinations of medical subject headings terms: (tumor [Title/Abstract]) OR (cancer [Title/Abstract]) AND (transcutaneous electrical acupoint stimulation [Title/Abstract]) AND (fatigue [Title/Abstract]) OR (depression [Title/Abstract]) OR (anxiety [Title/Abstract]). Manual hand-searching of reference lists and relevant papers was performed to identify additional studies or dissertations of relevance.

### 2.2. Inclusion and Exclusion Criteria

The inclusion criteria were as follows: (I) Studies involving adult (age >18 years) hospitalized patients with a cancer diagnosis based upon imaging or pathology [5]; (II) patients included were lucid without mental disorders; (III) studies involving the following intervention measures: the intervention group adopted TEAS whereas the control group adopted conventional nursing care or health education nursing method; (IV) primary study outcome was changes of CRF, and secondary outcomes were changes of negative emotions (depression or anxiety) and quality of life; and (V) study design was randomized controlled trials (RCTs). The exclusion criteria were as follows: (I) reviews or duplicate studies; (II) studies where the specific data could not be extracted; and (III) studies involving TEAS combined with other interventions in the intervention group.

### 2.3. Data Extraction

Two reviewers screened the search results by checking the titles and abstracts according to the inclusion criteria and subsequently read the full texts of the articles to select relevant studies. Data were independently extracted by two reviewers using the criteria outlined in the Cochrane Handbook for Systematic Reviews of Interventions [6]. The form includes four domains: (I) a description of the characteristics of the included studies (year of publication, name of the first author, study design); (II) characteristics of the participants (sample size, demographics, and disease information); (III) intervention (type and duration); and (IV) report results and relevant questionnaires. Disagreements between the two reviewers were resolved through discussion or consultation with a third member of the review team.

### 2.4. Quality Assessment

The Cochrane Collaboration Risk of Bias criteria were used to assess the risk of bias for each included study [7]. The following seven domains were considered: random sequence generation, allocation concealment, blinding of participants and personnel, blinding of outcome assessors, incomplete outcome data, selective reporting, and other sources of bias. Studies that fully met these criteria were classified as “A” (high-quality), whereas those that met some of the above criteria were classified as “B” (medium quality). Studies that did not meet any of the above criteria were classified as “C” (low quality) and excluded from the analysis.

### 2.5. Statistical Analyses

The meta-analysis was conducted using RevMan software (Version 5.3; Cochrane Collaboration, Oxford, England). The mean difference (MD) or standardized mean difference (SMD) with a 95% confidence interval (CI) was used to calculate the effect size for continuous variables. The magnitude of interstudy heterogeneity was quantified using the Cochran *Q* test (test level is *α* = 0.1) and the I^2^ statistics. When *P* < 0.05 and *I*^2^ >50%, the random-effects model was used to measure heterogeneity; otherwise, the fixed-effects model was used, and subgroup analysis was conducted to detect the potential source of heterogeneity. Finally, the publication bias was qualitatively analyzed by the funnel plots and quantitatively by Egger's test.

## 3. Results

### 3.1. Overall Summary of Meta-Analyses

A total of 267 studies were initially identified. We excluded 120 duplicate articles, 23 case reports or reviews, 32 articles not eligible for inclusion, 60 articles not meeting primary endpoints, and 23 articles without specific data. Finally, nine articles were included in our models (three English articles and six Chinese articles). The identification and screening of studies are shown in the flow diagram (Figure 1).

### 3.2. Characteristics of the Included Studies

A total of nine RCTs published between 2009 and 2020 were included in this analysis. The studies reported data on a total of 924 patients with cancer, including 460 patients in the interventional group and 464 patients in the control group. The sample size of the included studies ranged from 60 to 127, and the intervention time ranged from 5 days to 8 weeks. Six studies assessed CRF endpoints with RPFS, four studies included an assessment of anxiety or depression using the Self-rating Anxiety Scale (SAS) and Self-rating Depression Scale (SDS), and three studies included an assessment of the quality of life based on The European Organization for Research and Treatment of Cancer Quality of Life Questionnaire-Core30 (EORTc QLQ-C30) and Functional Assessment of Cancer Therapy General (FACt-G). The detailed characteristics are summarized in Table 1 [3, 4, 8–14].

### 3.3. Evaluation of the Methodological Quality of the Studies

Eight RCT studies used the randomization method. One study only mentioned randomization without illustrating the specific method. Three RCTs mentioned allocation concealment. Participants were blinded in two studies, and assessors were blinded in five studies. No statistically significant heterogeneity was observed among the nine studies (Figure 2).

### 3.4. Effects of TEAS on CRF

Six RCTs [3, 4, 10-13] that assessed the effect of TEAS on CRF (I^2^ = 0%, *P* = 0.95) showed that the CRF of the intervention group was significantly lower than that of the control group (SWD = −0.83, 95% CI: −0.99 to −0.66, *P* < 0.05), as shown in Figure 3. The included studies were further analyzed according to whether the intervention duration exceeded 28 days. In cases where the duration of intervention was <28 days, the CRF in the intervention group was significantly lower than that of the control group (SWD = −0.88, 95% CI: −1.13 to −0.63, *P* < 0.05). Similarly, in studies with a duration of intervention ≥28 days, the CRF of the intervention group was also significantly lower than that of the control group (SWD = −0.79, 95% CI: −1.01 to −0.57, *P* < 0.05) (Figure 4). Subgroup analyses based on the sample size showed that statistical difference between the two groups can be observed regardless of whether the sample size was >100 (SWD = −0.92, 95% CI: −1.25 to −0.59, *P* < 0.05) or ≤100 (SWD = −0.80, 95% CI: −0.99 to −0.60, *P* < 0.05) (Figure 4).

### 3.5. Effects of TEAS on Negative Emotions

Four RCTs [8–10, 14] assessed the effect of TEAS on negative emotions in patients with cancer (I^2^ = 93%, *P* < 0.05). The negative emotion in the intervention group was less severe than that in the control group (SWD = −1.46, 95% CI: −2.15 to −0.77, *P* < 0.05) (Figure 5). The analysis showed that there was a statistical difference between the two groups after intervention in terms of anxiety (SWD = −1.37, 95% CI: −2.34 to −0.40, *P* < 0.05) and depression (SWD = −1.64, 95% CI: −2.40 to −0.89, *P* < 0.05) (Figure 5).

### 3.6. Effects of TEAS on the Quality of Life

Three RCTs [11–13] assessed the impact of TEAS on the quality of life of patients with cancer (I^2^ = 83%, *P* < 0.05). The result showed that the quality of life in the intervention group was higher than that in the control group (SWD = 0.74, 95% CI: 0.20 to 1.27, *P* < 0.05) (Figure 6).

### 3.7. Publication Bias

The funnel plots of CRF and negative emotion were not suggestive of publication bias as indicated by relative symmetry about the cumulative effect size (Figures 7 and 8).

## 4. Discussion

In this meta-analysis, we examined the effects of TEAS on the CRF, anxiety, depression, and quality of life in cancer patients and found that TEAS significantly improved the CRF, anxiety, depression, and quality of life in cancer patients.

We focused on the most common symptoms related to TEAS in nine studies with cancer patients, namely, CRF, anxiety, and depression. CRF is one of the most common symptoms of cancer survivors, and it is estimated that up to 90% and 27–82% of patients suffer from CRF during and after cancer treatment, respectively [15, 16]. CRF is defined as multidimensional and distressing fatigue related to cancer and/or cancer treatment that interferes with activities of daily living and significantly diminishes the quality of life [17]. Although chemotherapy and radiation therapy can be effective in treating physical disorders, they can hardly improve mental health. In fact, anxiety, stress, and depression often occur before and during cancer treatment [18]. As shown in our meta-analysis, TEAS can effectively reduce CRF; however, it must also be acknowledged that considerable heterogeneity exists between studies, including different tumor types, duration of intervention, and sample size. It has already been suggested that TEAS can reduce levels of inflammatory cytokines and improve CRF, which is a common and persistent adverse reaction of cancer treatment [3, 19].

Our results are consistent with the findings of several RCTs [8–10, 14], indicating that TEAS can significantly reduce anxiety and depressive symptoms in patients with cancer. A variety of treatments can negatively affect cancer patients, leading to anxiety and depression symptoms [20]. Thoughtful application of TEAS can actually increase self-esteem and self-confidence, relieve discomfort, and alleviate anxiety and depression symptoms among cancer patients. In addition, our analysis showed that TEAS could significantly improve the quality of life of cancer patients. Nevertheless, our review found only three RCTs addressing the impact of TEAS on the quality of life of cancer patients. Taken together, the impact of TEAS on the quality of life of cancer patients is highly heterogeneous, partly due to different sample sizes, assessment scales, and others.

To the best of our knowledge, this is the first meta-analysis to investigate the effects of TEAS on CRF and negative emotions in patients with cancer. The quantitative evaluation of TEAS in our analysis can help strengthen the reliability of results and provide guidance for the clinical rehabilitation of cancer patients. Nevertheless, our study suffers from several limitations. First, our analysis was restricted to studies published in English or Chinese. Second, the review only analyzed a few studies with a small sample size.

## 5. Conclusions

In conclusion, TEAS can reduce CRF, anxiety, and depression and improve the quality of life of cancer patients. Given the above limitations, the current results should be interpreted with caution, and high-quality RCTs with larger sample sizes are warranted in the future to study the impact of TEAS on cancer patients.

## Figures and Tables

**Figure 1:** Study flow diagram.

**Figure 2:** Risk of bias graph.

**Figure 3:** Forest plot. Subgroup analysis of cancer-related fatigue in the interventional and control groups (intervention time). SD, standard deviation; CI, confidence interval.

**Figure 4:** Forest plot. Subgroup analysis of cancer-related fatigue in the interventional and control groups (sample size). SD, standard deviation; CI, confidence interval.

**Figure 5:** Forest plot. Subgroup analysis of negative emotions in the interventional and control groups (anxiety and depression). SD, standard deviation; CI, confidence interval.

**Figure 6:** Forest plot. Subgroup analysis of quality of life in the interventional and control groups. SD, standard deviation; CI, confidence interval.

**Figure 7:** Funnel plots of studies with cancer-related fatigue as the endpoint. SE, standard error; SMD, standardized mean difference.

**Figure 8:** Funnel plots of studies with negative emotions as the endpoint. SE, standard error; SMD, standardized mean difference.

**Table 1:** Characteristics of the included studies.

Author, year	Sample size (n, T/C)	Age (years) (mean ± SD or range)	Gender (F/M)	Cancer type	Treatment method	Intervention time	Outcome indicator (scale)	Quality
Tai et al., 2020 [8]	127, 62/65	–	–	Metastatic cancer	Surgery + chemotherapy	5 days	Anxiety (SAS)	B
Gao and Luo, 2019 [9]	84, 42/42	T: 40–74; C: 41–75	T: 19/23; C: 18/24	Lung cancer	Chemotherapy	8 days	Anxiety (SAS); depression (SDS)	B
Hu et al., 2019 [10]	100, 50/50	T: 65.24 ± 8.45; C: 64.70 ± 9.65	T: 18/32; C: 18/32	Lung cancer	Chemotherapy	21 days	CRF (RPFS); anxiety (SAS); depression (SDS)	B
Huang and Zhao, 2019 [11]	120, 60/60	T: 58.25 ± 6.91; C: 59.13 ± 7.62	T: 29/31; C: 32/28	Uncertain	Surgery + chemotherapy	8 weeks	CRF (RPFS); quality of life (EORTc QLQ-C30)	B
Li et al., 2020 [12]	108, 55/53	T: 59.85 ± 10.34; C: 56.83 ± 11.06	T: 28/27; C: 25/28	Uncertain	Chemotherapy	5 days	CRF (RPFS); quality of life (FACT-G)	B
Wu et al., 2017 [13]	113, 57/56	T: 58.53 ± 8.42; C: 58.52 ± 10.65	T: 15/42; C: 10/46	Lung cancer	Chemotherapy	28 days	CRF (RPFS); quality of life (EORTc QLQ-C30)	B
Hou et al., 2017 [3]	113, 57/56	T: 58.06 ± 8.42; C: 58.27 ± 10.57	T: 15/42; C: 10/46	Lung cancer	Chemotherapy	28 days	CRF (RPFS)	B
Sun, 2011 [4]	60, 30/30	T: 58.0 ± 6.1; C: 57.4 ± 6.9	T: 16/14; C: 18/12	Gastrointestinal cancer	Chemotherapy	7 days	CRF (RPFS)	B
Hu et al., 2017 [14]	113, 51/62	T: 59.98 ± 8.51; C: 58.81 ± 10.50	T: 15/36; C: 11/51	Lung cancer	Chemotherapy	28 days	Anxiety (SAS)	A

Undetermined in cancer type refers to the original literature indicating the inclusion of patients with unspecified tumor types. Full compliance with the risk of bias in the Cochrane RCTs is grade “A” (high-quality), and partial compliance with the original studies is grade “B” (moderate quality). *T*, interventional group; C, control group; F, female, M, male; CRF, cancer-related fatigue; RCT, randomized controlled trial; SAS, Self-rating Anxiety Scale; RPFS, Revised Piper Fatigue Scale; SD, standard deviation; SDS, Self-rating Depression Scale; EORTc QLQ-C30, European Organization for Research and Treatment of Cancer Quality of Life Questionnaire-Core 30.

## Data Availability

The datasets used and analyzed during the current study are available from the corresponding author upon reasonable request.
